The article "Artificial Bee Colony Based Gabor Parameters Optimizer (ABC-GPO) for Modulation Classification" was retracted in 2023. Reasons: signs of a paper mill; suspected computer-generated content; unreliable results or conclusions; concerns about the data.

# Artificial Bee Colony Based Gabor Parameters Optimizer (ABC-GPO) for Modulation Classification

**DOI:** 10.1155/2022/9464633

**Published:** 2022-09-30

**Authors:** Saad AlJubayrin, Mubashar Sarfraz, Sajjad A. Ghauri, Muhammad Rizwan Amirzada, Teweldebrhan Mezgebo Kebedew

**Affiliations:** ^1^Department of Computer Science, College of Computing and Information Technology, Shaqra University, Shaqra, Saudi Arabia; ^2^Faculty of Engineering and Computer Science, National University of Modern Languages, Islamabad, Pakistan; ^3^School of Engineering & Applied Sciences, ISRA University, Islamabad, Pakistan; ^4^Ethio Telecom, Addis Ababa, Ethiopia

## Abstract

Modulation classification is one of the essential requirements in the various cognitive radio applications where prior information about the incoming signal is unknown. The modulation classification using a pattern recognition approach can be achieved in 2 modules: first, parameters are extracted from the noisy signal, and then feature selection is carried out using a Gabor filter network (GFN). In the second module, features are exploited for classification purposes. The modulation formats considered for the purpose of classification are BPSK, QPSK, 8PSK, 16PSK, 64PSK, 4FSK, 8FSK, 16FSK, QAM, 8QAM, 16QAM, 32QAM, and 64QAM. The Gabor filter parameters and weights of the adaptive filter are attuned using the Delta rule and recursive least square (RLS) algorithm until the cost function is minimized. In the end, the artificial bee colony (ABC) algorithm is used to optimize the Gabor parameters as well as the classifier's performance. The simulation results show the supremacy of the proposed classifier structure.

## 1. Introduction

Automatic digital modulation classification (ADMC) is to classify the modulation format of the received signal, which has undergone channel effects and noise. For commercial and military communication systems, classification and identification of the modulation format are a significant phase formerly the demodulation at the receiver side. Rapid growth in the commercial wireless communication system demands adaptive, efficient spectrum access algorithms. Software-defined radio (SDR) and later, cognitive radio (CR) are examples of civilian adaptive structures [1–4].

Due to a lack of prior knowledge of the modulation format, ADMC becomes more complex and challenging. The modulation format includes modulation type, symbol duration, frequency deviation, carrier frequency/phase offsets, noise variance, channel amplitude, and so on. In Figure 1, a typical block diagram of ADMC is shown. The input symbols are first modulated and passed through a channel that adds the additive white Gaussian noise. At the receiver end, the first received signal is preprocessed; demodulation of the received signal and detection of the transmitted signal (information-bearing symbols) are executed after the modulation format is classified [5–7].

### 1.1. Contribution of the Article

The literature review shows that the choice of efficient features and classifier needs to be addressed for performance improvement in the classifier structure. Under the effect of fading channels and AWGN, GFN features for classification of modulation formats BPSK, QPSK, 8PSK, 16PSK, 64PSK, 4FSK, 8FSK, 16FSK, QAM, 8QAM, 16QAM, 32QAM, and 64QAM are presented in this paper. The classifier performance is further optimized by using the artificial bee colony algorithm (ABC). The performance of the proposed algorithm is evaluated with and without optimization.

### 1.2. Organization of the Article

The rest of the paper is as follows: section 2 contains a comprehensive review of the literature on automatic digital modulation classification. A system model with a proposed classifier structure is explained in section 3. The Gabor filter structure for digital modulation classification and the training and testing of the proposed algorithm are also presented in section 4. The detailed simulation results are carried out in section 4, which shows the supremacy of the proposed classifier. section 5concludes the paper.

## 2. Related Work

The ADMC can be generally classified into two categories: the likelihood ratio-based decision-theoretic approach and the feature extraction-based pattern recognition approach [8]. In a decision-theoretic approach, the decision is made based on the likelihood function (LF) of the received signal. Once the likelihood function is constituted, the latter classifies the modulation format of the received signal. The process of ADMC in the decision-theoretic approach may be viewed as multiple hypothesis tests or a sequence of pairwise multiple hypothesis tests. To compute the unconditional likelihood, the following are the well-known algorithms in the literature: average likelihood ratio test (ALRT), generalized likelihood ratio test (GLRT), hybrid likelihood ratio test (HLRT), and quasi-hybrid likelihood ratio test (QHLRT) [9–12].

Some related work for the decision-theoretic approach is presented in [13], where the authors use it to determine the modulation format for software-defined radio. A lookup table (LUT)-based classifier is proposed. In [14], only amplitude modulation formats are considered, and the proposed classifier is based on a hybrid maximum likelihood approach. In [15], likelihood algorithms (HLRT, QHLRT) are explored for digital modulation classification. The complexity of HLRT is evaluated, and whether QHLRT provides a reasonable solution is also discussed. The Cramer-Rao upper bound for BPSK and QPSK modulation formats is also employed. In [16], the authors survey the existing techniques for the modulation classification problem.

Feature extraction-based pattern recognition approaches are suboptimal. The FB approach is carried out in two modules, feature extraction and classifier structure [17]. The features extracted are spectral features, statistical features, cyclo-stationary features, and time-frequency features. They are found in the literature for the FB approach. The features extracted from the PSO-SC with the best clustering radius are shown in [18]. The spectral features are used to classify the 9 analogue and digital modulation formats, and the back propagation neural network is used as a classifier in [19, 20]. The proposed algorithm in [21] uses genetic programming with K-nearest neighbour (GP-KNN) and higher-order cumulants as features to classify the four modulation formats.

A fuzzy logic-based modulation classification is proposed in [22]. The author develops a nonsingleton fuzzy logic classifier by using a fuzzy logic system (FLS). In [23], the author proposed cyclo-stationary-based feature detection for the problem of modulation classification for cognitive radios. The author employed a neural network (NN) and hidden Markov model (HMM)-based classifiers. The spectral features are developed for the classification of ASK, PSK, and FSK using a maximum likelihood decision-based criterion as a classifier [24]. In [25], the author utilises the higher-order cumulants (HOC) as features, and the classifier is based on a support vector machine (SVM). The binary SVM and multiclass SVM are used in conjunction with genetic algorithms, and classifier performance is evaluated with and without optimization.

The spectral features and HOC are extracted, and two multilayer perceptron recognizers, namely a back propagation neural network (BPNN) and resilient backpropagation (RPROP), are used in [26]. The bee's algorithm for optimization of the performance of the classifier is utilised in [27]. The features used are HOC and instantaneous characteristics of digital modulations. The hierarchical SVM is used as a classifier. Under the multipath fading environment, the normalised fourth-order cumulants are used to classify the BPSK, QPSK, and QAM. The Cramer–Rao lower bound is consequent to the features in [28]. The extracted time frequency is used as input to an MLP-based NN for the classification of digital modulation formats in [29, 30].

## 3. Proposed Classifier Structure

### 3.1. System Model

The generalized expression for the received signal is given as follows:

(1) $$\begin{array}{c} r\left(n\right)=\overset{L}{\underset{l=0}{\sum }}h\;\left[n,l\right]x\left[n-l\right]+w\left(n\right), \end{array}$$

where, *L* is the order of Multipath channel, *x*(*n*) is the modulated signal, *w*(*n*) is the additive white Gaussian noise, and h[n,l] is the response of the channel. In a matrix form, the following equation is given as follows:

(2) $$\begin{array}{c} r_{n}=H_{n}x_{n}+w_{n}. \end{array}$$

Table 1 shows the symbols and their descriptions, which are used in the article. The system model of proposed classifier structure, which is an artificial bee colony assisted Gabor filter is shown in Figure 2. The proposed classifier structure classifies the BPSK, QPSK, 8PSK, 16PSK, 64PSK, 4FSK, 8FSK, 16FSK, QAM, 8QAM, 16QAM, 32QAM, and 64QAM efficiently.

### 3.2. Gabor Filter Structure

The Gabor filter-based architecture is a tool for efficient feature extraction from the received signal. The Gabor atom is defined as follows in [31]:

(3) $$\begin{array}{c} g_{i}\left(t\right)=\frac{1}{\sqrt{\sigma_{i}}}e^{-\pi {\left(t-c_{i}/\sigma_{i}\right)}^{2}}\cos\left(f_{i}t\right), \end{array}$$

where, *c*, *σ* and *f* are the shift, scale, and modulation parameters, respectively. The output of the *i*^*th*^ Gabor atom node is corresponding to the received signal is given as follows:

(4) $$\begin{array}{c} \phi_{i}=\left|r_{i}\underset{g_{i}\left(t\right)}{\underset{⏟}{\frac{1}{\sqrt{\sigma_{i}}}e^{-\pi {\left(t-c_{i}/\sigma_{i}\right)}^{2}}\cos\left(f_{i}t\right)}}\right|. \end{array}$$

The GFN output *ϕ*_*i*_ in the input layer is weighted by *w*_*i*_ i.e.

(5) $$\begin{array}{c} y\left(n\right)={\sum^{}}_{i=1}^{M}\phi_{i}w_{i}. \end{array}$$

The difference between the desired response *d*(*n*) and the output *y*(*n*) is the error function denoted by the following equation:

(6) $$\begin{array}{c} e\left(n\right)=d\left(n\right)-y\left(n\right). \end{array}$$

The extracted features *c*, *σ* and *f* are the Gabor atom parameters and weights of the adaptive filter *w* are adjusted until the cost function is minimized. The cost function is the sum of squared errors, which is [31]given as follows:

(7) $$\begin{array}{c} J\left(n\right)={\left[e\left(n\right)\right]}^{2}. \end{array}$$

### 3.3. Training of the Classifier

Figure 3 shows the training process for ADMC. The two adaptive algorithms are executed by the Gabor filter network in the training phase of ADMC; features are obtained by adjusting the Gabor atom parameters (*c*, *σ* and *f*) for each modulation format in the first algorithm, while in the second algorithm the weights are adjusted to minimize the error function. The delta rule, which is used to update the parameters of GFN, is taken from [31].The updating of shift, scale, and frequency parameters are shown in equations (8)–(10).

(8) $$\begin{array}{c} \begin{array}{c} c_{i}\left(n+1\right)=c_{i}\left(n\right)+\eta_{c}\left(d\left(n\right)-y\left(n\right)\right)w_{i}\times \\ \left[\frac{x_{i}}{\sqrt[{5}]{\sigma_{i}}}\cos\left(f_{i}t\right)2\pi \left(t-c_{i}\right)e^{-\pi {\left(t-c_{i}/\sigma_{i}\right)}^{2}}\right] \end{array}, \end{array}$$

(9) $$\begin{array}{c} \begin{array}{c} \sigma_{i}\left(n+1\right)=\sigma_{i}\left(n\right)+\eta_{\sigma }\left(d\left(n\right)-y\left(n\right)\right)w_{i}\times \\ \left[\frac{x_{i}\cos\left(f_{i}t\right)}{\sqrt{\sigma_{i}}}e^{-\pi {\left(t-c_{i}/\sigma_{i}\right)}^{2}}\left[\frac{2\pi {\left(t-c_{i}\right)}^{2}}{\sigma^{2}}-\frac{1}{2\sigma_{i}}\right]\right] \end{array}, \end{array}$$

(10) $$\begin{array}{c} \begin{array}{c} f_{i}\left(n+1\right)=f_{i}\left(n\right)+\eta_{\sigma }\left(d\left(n\right)-y\left(n\right)\right)w_{i}\times \\ \left[-\frac{t}{\sqrt{\sigma_{i}}}x_{i}e^{-\pi {\left(t-c_{i}/\sigma_{i}\right)}^{2}}\sin\left(f_{i}t\right)\right] \end{array}. \end{array}$$

The weights of the GFN are updated using an RLS filter, and the weight updating equation is shown in equation (13)

(11) $$\begin{array}{c} k\left(n\right)=\frac{k\left(n-1\right)\Phi \left(n\right)}{\lambda +\Phi^{T}\left(n\right)K\left(n-1\right)\Phi \left(n\right)}, \end{array}$$

(12) $$\begin{array}{c} w\left(n\right)=w\left(n-1\right)+k\left(n\right)e\left(n\right). \end{array}$$

### 3.4. Testing of the Classifier

In the testing phase of the proposed classifier structure, the received signal is first serially converted to parallel and then fed to the trained Gabor filter bank. The error has been calculated for each Gabor filter as shown in Figure 4. The minimum error corresponds to the desired modulation format [31].

### 3.5. Artificial Bee Colony Optimizer

The artificial bee colony (ABC) algorithm is used to optimize the Gabor filter parameters (*c*_*i*_, *sigma*_*i*_, *f*_*i*_) as well as the weights *w*(*n*). The Gabor parameters and weights are optimized by minimizing the cost function defined in (7). The (*c*, *σ*, *f*, *w*) are randomly initialized at the start of the algorithm, and fitness is evaluated. The ABC optimization adapts to the natural behaviour process of the honeybees. The solutions are updated by searching the neighbouring areas through three different processes that are carried out by employer bees, onlooker bees, and scout bees. Algorithm 1 presents the brief steps for the ABC-GPO algorithm.

## 4. Experimental Classification Results and Analysis

The performance of the proposed classifier using the optimized Gabor filter features is evaluated in this section. The thirteen modulation formats are considered for classification, i.e., BPSK, QPSK, 8PSK, 16PSK, 64PSK, 4FSK, 8FSK, 16FSK, QAM, 8QAM, 16QAM, 32QAM, and 64 QAM. For simplicity, these modulated signals are replaced by P1, P2, P3, P4, P5, P6, P7, P8, P9, P10, P11, P12, and P13. All the simulations are done in MATLAB R2020a. The performance metric is the percentage classification accuracy (PCA). A total of 100000 realizations have been taken with 1024 no. of samples. The data set has been divided into training, validation, and testing samples, i.e., 80%, 10%, and 10%.

### 4.1. PCA on AWGN Channel

Figure 5 shows the training and testing performance of the classifier on the AWGN channel for all considered modulation formats. The training of the proposed GFN is carried out at different SNRs. The percentage classification accuracy for the training and testing of the classifier is approximately 90% at an SNR of −5 dB. At 10 dB SNR, the classification accuracy approaches 100% for the training and testing of a classifier. The total number of samples taken is 1024, with 10,000 realizations.

### 4.2. PCA on Rician Channel

Figure 6 shows the training and testing performance of the classifier on the Rician fading channel with AWGN. The percentage classification accuracy for the training and testing of the classifier is approximately 99.42% and 98.50% at an SNR of 10 dB, respectively, which is relatively low as compared to the AWGN channel, while PCA is below 90% at −5 dB of SNR.

### 4.3. PCA on Rayleigh Channel

Figure 7 shows the training and testing performance of the classifier on the Rayleigh fading channel with AWGN. The percentage classification accuracy for the training and testing of the classifier is approximately 96.75% and 94.98% at an SNR of 10 dB, respectively, while the classification accuracy for testing is approximately 80% at −5 dB of SNR.

### 4.4. Optimized PCA on AWGN Channel

Figure 8 shows the training performance comparison with and without optimization in the presence of additive white Gaussian noise. The PCA is far better for the optimized Gabor features-based classification as compared to the nonoptimized Gabor feature classifier. The training accuracy of the optimized classifier is approximately 100% at an SNR of 5 dB, while the nonoptimized Gabor features-based classifier is approaching 100% at 8 dB of SNR. The quantitative improvement in the classification accuracy is about 4.4% at −5 dB of SNR.

The testing classification of optimized and nonoptimized Gabor features-based classification is shown in Figure 9. The PCA is much better compared to the nonoptimized-based classifier. As it is clear from Figure 9, the PCA for optimized and nonoptimized Gabor features is 99.96% and 98.87%, respectively. The quantitative improvement in the testing accuracy at −5 dB of SNR is greater, i.e., around 4%.

Table 2 shows the confusion matrix for the classification of digital modulation formats using Gabor features without optimization. The classification accuracy shown in the diagonal is approximately 97.84% for the case of the AWGN channel. From the confusion matrix, the Gabor features are capable of classifying the considered modulation formats with high accuracy under the effect of white Gaussian noise.

Table 3 shows the confusion matrix for the classification of digital modulation formats using optimized Gabor features. The classification accuracy shown in the diagonal is approximately 99.45% for the case of the AWGN channel at 8 dB of SNR.

### 4.5. Comparison with State of Art Existing Techniques

Table 4 shows the method proposed and the year, the number of modulation formats to be classified, the percentage classification accuracy at a SNR of 10 dB, and the number of features extracted from the received signal. With the existing techniques, modulation formats considered for classification are in fewer numbers and the number of features used is greater, and classification accuracy is also not above 90% for the maximum cases. The efficient features that we extracted are only three, and we successfully classified thirteen modulation formats at an SNR of 3 dB.

### 4.6. Complexity Analysis

The algorithm requires time and memory resources to perform the computations, and the number of required resources determines the computational complexity of the algorithm. The proposed algorithm runs in two sections: the GFN and the ABC algorithm. The computational complexity is separate for GFN with or without optimization. The complexity of the proposed algorithm without optimization is the complexity of the GFN, which is given in [40]as follows:

(13) $$\begin{array}{c} O_{GFN}=O\left(N\log N\right), \end{array}$$

where *N* is the number of samples, however, the complexity of the proposed algorithm with optimization is as follows:

(14) $$\begin{array}{c} O_{ABC-GFN}=O\left(Iterations*No.ofBees*eq.\left(7\right)\right). \end{array}$$

## 5. Conclusion

The automatic digital modulation classification using GFN is considered in this research article. The extracted features are GF features for the considered BPSK, QPSK, 8PSK, 16PSK, 64PSK, 4FSK, 8FSK, 16FSK, QAM, 8QAM, 16QAM, 32QAM, and 64QAM modulation formats. The bee colony algorithm is used to optimize the algorithm's results. The simulation results show the performance of the classifier with and without optimization of the algorithm. The performance fading channels is compared to the state of the art of existing techniques.

## Figures and Tables

**Figure 1:** Typical block diagram of ADMC.

**Figure 2:** System model.

**Figure 3:** Training structure of the Gabor filter for ADMC.

**Figure 4:** Testing of proposed classifier.

**Figure 5:** Training and testing of the proposed classifier on the AWGN model.

**Figure 6:** Training and testing of the proposed classifier on the Rician model.

**Figure 7:** Training and testing of the proposed classifier on the Rayleigh model.

**Figure 8:** Training of the proposed classifier with/without optimization.

**Figure 9:** Testing of the proposed classifier with/without optimization.

**Algorithm 1:** ABC-based Gabor parameters optimizer (ABC-GPO).

**Table 1:** Symbols and description.

Symbol	Description
*L*	Order of multipath channel
*g*_*i*_(*t*)	Gabor atom
*σ*_*i*_	*i* ^*th*^ Gabor scale parameter
*c*_*i*_	*i* ^*th*^ Gabor shift parameter
*f*_*i*_	*i* ^*th*^ Gabor modulation parameter
*k *(*n*)	Gain vector
*K *(*n*)	Weight error correlation
Φ(*n*)	Time average correlation matrix
*λ*(*n*)	Positive constant

**Table 2:** Percentage classification performance of ADMC at SNR of 8 dB without optimization.

	*P*1	*P*2	*P*3	*P*4	*P*5	*P*6	*P*7	*P*8	*P*9	*P*10	*P*11	*P*12	*P*13
*P*1	99												
*P*1		96											
*P*1			97										
*P*1				96									
*P*1					97								
*P*1						98							
*P*1							97						
*P*1								98					
*P*1									96				
*P*1										97			
*P*1											98		
*P*1												97	
*P*1													98

**Table 3:** Percentage classification performance of ADMC with optimization at a SNR of 8 dB.

	*P*1	*P*2	*P*3	*P*4	*P*5	*P*6	*P*7	*P*8	*P*9	*P*10	*P*11	*P*12	*P*13
*P*1	100												
*P*1		99											
*P*1			98.5										
*P*1				98.8									
*P*1					99.2								
*P*1						99.1							
*P*1							99.6						
*P*1								99.4					
*P*1									98.4				
*P*1										99.1			
*P*1											99.4		
*P*1												98.4	
*P*1													98.8

**Table 4:** Comparison with the existing techniques.

Method and reference	Number of modulation	Classification accuracy in % at SNR = 10 dB	No. of features
Pdf of the received signal, zero crossing [32]	PSK, FSK (7)	98 (15 dB of SNR)	4
Spectral features [33]	PSK, FSK (6)	90	5
Spectral features and moments [34]	PSK, FSK (9)	96 (15 dB of SNR	9
Constellation shape [35]	PSK, QAM (3)	90 (5 dB of SNR	4
HOC [36]	PSK, QAM (8)	96	2
Neural networks [37]	PSK, FSK, QAM (7)	93 (8 dB of SNR)	5
Back propagation (BP) algo., resilient BP algo [26]	PSK, FSK, QAM (10)	89.96, 99.95	17
Time frequency features [29]	FSK, PSK (6)	97.64	4
Normalized cummulants [28]	PSK, QAM (5)	97.5	1
Cummulants features, multiclass SVM [25]	PSK, QAM (9)	97.56	12
Spectral features and moments [30]	FSK, QAM (12)	99.95	8
HOC and spectral features, multiclass SVM [27]	PSK, QAM, FSK (11)	97.45	11
Gabor filter based features [31]	PSK, FSK, QAM (18)	100	3
HOC and SVM [38]	QAM (6)	98.7 (5 dB of SNR)	11
HOC and polynomial classifier [39]	PSK (5)	98	10
Proposed optimized classifier	PSK, FSK, QAM (13)	100 (8 dB of SNR)	3

## Data Availability

This article does not meet the criteria for data sharing since no datasets were generated or analyzed.
